The article "Classification of Benign and Malignant Lung Nodules Based on Deep Convolutional Network Feature Extraction" was published in 2021. Journal: J Healthc Eng.

# Classification of Benign and Malignant Lung Nodules Based on Deep Convolutional Network Feature Extraction

**DOI:** 10.1155/2021/8769652

**Published:** 2021-10-27

**Authors:** Enhui Lv, Wenfeng Liu, Pengbo Wen, Xingxing Kang

**Affiliations:** ^1^School of Medical Information & Engineering, Xuzhou Medical University, Xuzhou 221004, China; ^2^Department of Information Center, Weihai Ocean Vocational College, Rongcheng 264300, China

## Abstract

With the rapid development of detection technology, CT imaging technology has been widely used in the early clinical diagnosis of lung nodules. However, accurate assessment of the nature of the nodule remains a challenging task due to the subjective nature of the radiologist. With the increasing amount of publicly available lung image data, it has become possible to use convolutional neural networks for benign and malignant classification of lung nodules. However, as the network depth increases, network training methods based on gradient descent usually lead to gradient dispersion. Therefore, we propose a novel deep convolutional network approach to classify the benignity and malignancy of lung nodules. Firstly, we segmented, extracted, and performed zero-phase component analysis whitening on images of lung nodules. Then, a multilayer perceptron was introduced into the structure to construct a deep convolutional network. Finally, the minibatch stochastic gradient descent method with a momentum coefficient is used to fine-tune the deep convolutional network to avoid the gradient dispersion. The 750 lung nodules in the lung image database are used for experimental verification. Classification accuracy of the proposed method can reach 96.0%. The experimental results show that the proposed method can provide an objective and efficient aid to solve the problem of classifying benign and malignant lung nodules in medical images.

## 1. Introduction

Lung cancer is one of the most common cancers in the world. Compared with other cancers, there are no obvious symptoms at an early stage. Early detection of lung cancer in its nodular form, screening, classification, and medical management have been demonstrated to be extremely helpful and effective in decreasing lung cancer mortality [1]. Therefore, how to effectively diagnose lung nodules has become a topic of primary concern. The detection and diagnosis of lung nodules can be achieved by imaging procedures, such as CT imaging [2], magnetic resonance imaging [3], etc. The diagnosis of suspected lung nodules remains difficult due to human subjectivity, fatigue, and other limitations related with CT images. In some cases, radiologists may not be able to identify some nodules with diameters <3 mm [4]. Therefore, it is important to study the method of classifying benign and malignant lung nodules in a computer-aided diagnosis (CAD) system for early detection and diagnosis of lung cancer.

The article "Classification of Benign and Malignant Lung Nodules Based on Deep Convolutional Network Feature Extraction" was published in 2021. Journal: J Healthc Eng.

At present, the classification of benign and malignant lung nodules in the CAD system is mainly performed by extracting the underlying features of the CT image of lung nodules, such as the shape, position, texture, and density, through machine learning methods [5]. Moreover, this classification method based on the underlying features has obtained good results in improving the accuracy of lung nodule diagnosis and reducing the labor intensity of doctors. However, the real nodule shape, size, and texture features are highly variable. And the extraction of the underlying features is generally based on manual design, thus failing to fully describe these real nodules, resulting in a low correct rate of overall detection results [6]. Therefore, how to perform automatic feature extraction and selection on CT images of lung nodules has become a hot topic of research.

In recent years, with the rapid development of deep learning, many studies have also demonstrated that convolutional neural networks (CNN) can be well applied to the field of medical images [7–10]. This is mainly because CNN, as an end-to-end network architecture, can automatically extract features from the input image. In the classification of lung nodules, the commonly used CNN models are the two-dimensional CNN (2D-CNN) and the three-dimensional CNN (3D-CNN). Shen et al. [11] proposed a hierarchical learning framework multiscale CNN (MCNN) for lung nodule classification by extracting discriminatory features from alternating stacked layers to capture the heterogeneity of lung nodules. This network not only improves the classification accuracy, but also has strong robustness to noisy input. It is worth noting that the network architecture of MCNN consists of alternating stacks of convolutional and max-pooling layers, and takes a long time to extract features. Therefore, Tran et al. [12] proposed a new deep learning method to improve the classification accuracy of lung nodules in CT. The central idea is as follows: firstly, a novel 15-layer 2D-CNN architecture is constructed to automatically extract lung nodule features and classify them as nodules or non-nodules. Then, the focal loss function is used for network training to improve the classification accuracy of the model. However, with the increment of network depth, network training problems may occur, such as overfitting [13] and gradient vanishing [14]. The information behind the network is not well fed back due to deeper network depth, which results in network performance degradation. Therefore, the residual network solves the gradient dispersion due to network deepening by generating residual blocks to fit the original function [15]. Based on this study, Nibali et al. [16] achieved 89.9% accuracy in lung nodule classification on the LIDC dataset by constructing a fully convolutional residual neural network, which not only fully exploited the shallow and deep features of lung nodule images, but also reduced the number of parameters. Abraham et al. [17] used three 2D-CNN (AlexNet, VGG16, and SilNet) to classify lung nodules and designed a new network model based on the obtained inference results to eliminate the deficiencies of existing networks for early prediction of lung cancer. Through the above study, it was found that 2D-CNN network has the advantages of low network complexity and fast computation, but it ignores some spatial information. This is mainly due to the fact that CT scans are 3D images, most existing CNN-based approaches use a 2D model, which cannot capture the spatial information between slices. Dou et al. [18] proposed a 3D-CNN for false positive in automated pulmonary nodule detection from CT scans. The experimental results show that compared with 2D-CNN, the 3D-CNN can encode richer spatial information and extract more representative features via their hierarchical architecture trained with 3D samples. At the same time, Fu et al. [19] developed a computer-aided lung nodule detection system using a three-dimensional deep CNN to make full use of three-dimensional spatial information. The system mainly includes two stages: lung nodule detection stage and classification stage. In particular, in the detection phase, an 11-layer 3D fully CNN is used for the first time to screen all lung nodules. Experimental results demonstrate the effectiveness of using 3D deep CNNs for lung nodule detection. Zhao et al. [20] combined multiscale feature fusion with multiattribute classification to construct a new 3D-CNN model and proposed a new loss function to balance the relationship between different attributes, achieving a classification accuracy of 93.92% on the LIDC dataset. Gao and Nie [21] proposed a method to discriminate benign and malignant lung nodules by combining deep CNN with imaging features. The central idea is as follows: firstly, segment the lung nodule region from CT images and extract the imaging features of the nodule region using traditional machine learning methods. Then, train the 3D-Inception-ResNet model using the intercepted lung nodules, extract the CNN features learned by the network, combine the two types of features, and use the Random Forest (RF) model for feature selection. Finally, a Support Vector Machine (SVM) was used for the differential diagnosis of benign-malignant lung nodules. Zhang et al. [22] proposed a 3D dense network architecture by taking advantage of densely connected convolution, which encourages feature reuse and alleviates the vanishing gradient problem. The result shows that the proposed model has achieved good classification performance in the malignant suspiciousness of lung nodules and achieved 92.4% classification accuracy. Through the above research and analysis, it can be known that the classification effect of 3D-CNN is better owing to the full extraction of feature information, but it requires a large amount of data and takes a long time to calculate [23]. However, when the number of medical image datasets is small, training a 3D-CNN model from scratch will result in poor classification results. Moreover, the training algorithm of deep CNN usually adopts a layer-by-layer training mechanism based on gradient descent [24], where the network is trained layer by layer from the bottom up, and the output of the previous layer is used as the input of the next layer. The disadvantage of this learning mechanism is that the image pixels after the first layer are discarded, making the connection between the higher layers of the model and the input become sparser, which in turn causes the error correction signal to become smaller and smaller from the top layer down and tends to converge to a local minimum. In addition, when using the backpropagation algorithm to propagate the gradient, the network parameters cannot be learned effectively as the number of network layers deepens, resulting in the gradient dispersion [25].

The article "Classification of Benign and Malignant Lung Nodules Based on Deep Convolutional Network Feature Extraction" was published in 2021. Journal: J Healthc Eng.

Guided by the above studies and observations, we propose a novel deep convolutional network learning (DCN) method to obtain better performance in classifying benign and malignant lung nodules. The central idea is as follows: firstly, segment the lung nodule region from the lung CT images to obtain the lung nodule images and perform zero-phase component analysis (ZCA) whitening on the image data so that all features in the images have the same variance and low feature-to-feature correlation. Then, add a multilayer perceptron layer after each convolutional layer of the constructed DCN to achieve cross-channel information interaction and integration. Finally, obtain the second derivative information of the error function directly without calculating the Hessian matrix, and introduce a momentum coefficient based on this information to improve the convergence of the network. The key contributions are summarized as follows: (1) the use of ZCA whitening to process the input data can reduce the correlation between image pixels and thus eliminate redundant information; (2) by introducing multiple perceptron layers after each convolutional layer can further enhance the expression capability of the network; (3) the use of small batch random gradient descent with additional momentum coefficients to train the deep network can effectively avoid gradient dispersion and enhance the generalization capability of the network.

The article "Classification of Benign and Malignant Lung Nodules Based on Deep Convolutional Network Feature Extraction" was published in 2021. Journal: J Healthc Eng.

## 2. Materials and Methods

### 2.1. Network System Architecture

To use DCN to learn the features of CT images of lung nodules and enhance the representation of the model by introducing multilayer perceptron, which in turn improves the classification accuracy of lung nodule images. In addition, a momentum coefficient is introduced to improve the convergence in the minibatch stochastic gradient descent (MB-SGD) method to train the deep network model. The structural diagram of the lung nodule benign and malignant classification system based on DCN feature extraction is shown in Figure 1, which consists of three main parts. Stage I includes lung nodule image segmentation and extraction: firstly, a series of corresponding binary images are extracted from a large number of original lung CT images. Then, the binary image and the original image performed an “and” symbol operation to obtain the lung nodule images. Stage II is image preprocessing: redundant information among the lung nodule images extracted in Stage I is eliminated using ZCA whitening to reduce the correlation among the input image pixels. Stage III is DCN feature learning: firstly, the lung nodule images obtained from stage II processing are used as the input of the DCN. Then, a multilayer perceptron layer is introduced after each convolutional layer to realize cross-channel information interaction and integration. Finally, the MB-SGD method with a momentum coefficient is used to fine-tune the DCN to avoid the gradient dispersion problem.

### 2.2. Lung Nodule Image Segmentation and Extraction

To study early cancer detection in high-risk populations, the National Cancer Institute (NCI) published the Lung Image Database Consortium (LIDC) by collecting medical image files of the lung and corresponding lesion annotation of diagnostic results [23]. The LIDC dataset collected 1018 clinical lung CT scans, the size is 512 × 512, and each CT scan contained a relevant XML file containing the independent diagnostic results of four experienced radiologists [20]. Among them, radiologists marked 928 lung nodules, most of which were 3–30 mm in size. The diagnostic results include the coordinates of the lung nodules larger than 3 mm in diameter and the degree of malignancy. However, because of the small size of lung nodules, it is unrealistic to classify lung nodules by processing the whole image. Therefore, we need to extract the lung nodule areas based on the nodule center coordinate marked by the doctor in the XML file. In the LIDC dataset, radiologists quantified the malignancy of lung nodules on a scale of 1 to 5: neither likely, moderately unlikely, uncertain, moderately suspicious, and highly suspicious. When classifying benign and malignant levels, those with a level greater than or equal to 3 were classified as malignant, and those with a level less than 3 were classified as benign. There is variability in the marking of nodule locations by different experts, which results in the uniqueness of nodule areas. To eliminate the differences between experts and obtain standard lung nodule images, we use the threshold probability map (TPM) method to segment lung CT scans [26]. The central idea is as follows: firstly, according to expert experience, a weight value is set for each expert's annotation to indicate the reliability of the expert annotation. Then, each pixel in the lung nodule region marked by the expert is set to the same weight value. Finally, the weight value of the pixel is the sum of the weight values marked by all experts for the pixel. Now, assuming that the four experts have the same experience, the weight value of each expert is 0.25. If a pixel is marked as a component of a nodule by an expert, the probability that the pixel is a nodule is 0.25. If marked by 3 experts, the probability is 0.75. Thus, the lung nodule region is transformed into a mapping map with probability values between 0 and 1. When segmenting the lung nodule images, only a threshold T is set, and the pixels higher than T are set to 1, and the pixels lower than T are set to 0. This generates the corresponding binary images. Finally, this binary image is summed with the original image to obtain the lung nodule image. To improve the credibility of the study, when selecting lung nodule images in the LIDC dataset, we only considered cases in which at least three radiologists have made such a diagnosis of malignancy. Therefore, we segmented and extracted images of lung nodules, and eventually obtained a total of 750 cases of lung nodules, including 353 benign cases and 397 malignant cases. Due to the inconsistent size of lung nodules, to facilitate the learning and training of the DCN, they were normalized and transformed into grayscale images with a size of 28 × 28. The processed part of the sample image is shown in Figure 2.

The article "Classification of Benign and Malignant Lung Nodules Based on Deep Convolutional Network Feature Extraction" was published in 2021. Journal: J Healthc Eng.

### 2.3. Image Preprocessing

It is given that *I*={*I*^(1)^, ⋯, *I*^(*i*)^, ⋯, *I*^(*d*)^} ∈ *R*^*I*_*W*_×*I*_*H*_×*C*^ is a collection of *d* images of the size *I*_*W*_ × *I*_*H*_ and *C* denotes the channel of the image. First, because the visual images are highly affected by the light, to reduce the impact of image brightness on feature learning, the images are normalized for contrast [27] using the following equation:

(1) $$\begin{array}{c} q^{\left(i\right)}=\frac{I^{\left(i\right)}-\mathrm{mean}\left(I^{\left(i\right)}\right)}{\sqrt{\mathrm{var}\left(I^{\left(i\right)}\right)+\varepsilon }}, \end{array}$$

where mean(·) is the matrix averaging function. The normalization parameter *ε* is introduced to suppress the generation of experimental noise and prevent the denominator from being 0. For color image and grayscale image, *ε* is usually taken as 10.

Because of the strong correlation between adjacent pixels of the image, it contains a large amount of redundant information. To make all features in the image have the same variance and low feature-to-feature correlation, we perform ZCA whitening on the input data so that the whitened data is as close to the original data as possible with the same dimensionality. A matrix variation is performed for each image *q*^(*i*)^ in the image collection *Q*={*q*^(1)^, *q*^(2)^, ⋯, *q*^(*d*)^}, *q*^(*i*)^ ∈ *R*^*I*_*W*_×*I*_*H*_×*C*^ obtained by the contrast normalization operation, with the value of each image pixel point as an element to form *d* column vectors, each of length *I*_*W*_ × *I*_*H*_ × *C*, to form a *I*_*W*_ × *I*_*H*_ × *C*-row and *d*-column matrix of values Ψ. By performing an eigenvalue decomposition of the covariance matrix *C*=cov(Ψ), [*V*, *D*]=eig(*C*) is obtained, and then scaling the input data using the feature factors:

(2) $$\begin{array}{c} \Psi_{\mathrm{PCAwhite}}=\frac{\left(\Psi -\mathrm{mean}\left(\Psi \right)\right)\;•V}{\sqrt{\mathrm{diag}\left(D\right)+\xi }}, \end{array}$$

where *ξ* is the whitening factor. To avoid unstable values or data overflow due to eigenvalues diag(*D*) close to 0, *ξ* can be taken as a very small positive number. Based on this, ZCA whitening is performed using equation (3), and each column of the obtained matrix corresponds to the image data after ZCA whitening.

(3) $$\begin{array}{c} \Psi_{\mathrm{ZCAwhite}}=\Psi_{\mathrm{PCAwhite}}•V^{T}. \end{array}$$

### 2.4. DCN for Feature Learning

In the lung nodule image classification, the category of each image is described by two classifications of benign or malignant. Based on the guidance of the above study, we used DCN to extract all lung nodule images features and used a softmax-loss classifier for binary classification. The feature learning model based on DCN is shown in Figure 1. The model consists of an input layer, a feature extraction layer, and an output layer. The learning process is as follows: firstly, a feature map in the convolutional layer is generated by convolving the same convolutional kernel based on a weight sharing strategy to reduce model complexity and training parameters. Then, in the pooling layer, the features of the convolutional layer features are nonlinearly downsampled to filter out similar features, thereby reducing computational complexity and enhancing the invariance of local features. Finally, a softmax-loss classifier is used to build a multitask classifier for the learned deep features. Compared with other DCN, we achieve cross-channel information interaction and integration by adding multiple layers of perceptron layers in the network architecture, thus further enhancing the generalization ability of the deep network. In the actual construction process, the network architecture is equivalent to the introduction of two 1 × 1 convolutional layers, which only change the convolutional kernel size and have no effect on the feature map size.

The article "Classification of Benign and Malignant Lung Nodules Based on Deep Convolutional Network Feature Extraction" was published in 2021. Journal: J Healthc Eng.

Let the data of the lung nodule image after ZCA whitening be *X*={*x*^(1)^, ⋯, *x*^(*i*)^, ⋯, *x*^(*d*)^},  *x*^(*i*)^ ∈ *R*^*I*_*W*_×*I*_*H*_×*C*^. Since the preprocessed lung nodule images are grayscale images, the input data *x*^(*i*)^ and the convolution kernel are both 2D structures. The convolution layer convolves the input data or the previous layer feature map with multiple sets of convolution kernels, and then sums the corresponding positions of the output, adds the bias term, and obtains the convolution layer feature map under the action of the activation function. Its output feature map is calculated as follows:

(4) $$\begin{array}{c} x_{j^{\prime }}^{l}=f\left(\sum_{j\in M^{l}}x_{j}^{l-1}*f_{jj^{\prime }}^{l}\right), \end{array}$$

where *l* is the number of convolutional layers. *x*_*j*′_^*l*^ denotes the *j*′ output feature map of layer *l*. *f*_*jj*′_^ *l*^ is the convolution kernel connecting the *j* feature map of layer *l* − 1 with the *j*′ feature map of layer *l*. *M*^*l*^ is the number of feature maps in layer *l* − 1. *f*(·) denotes the nonlinear activation function ReLU. ^∗^ is the convolution operator. Due to the data distribution of the input, image will change after convolution operation, which leads to the internal covariance shift problem [28]. Therefore, we correct the data distribution by introducing a BN layer in the network architecture. The data after BN processing is equivalent to PCA dimensionality reduction [29]; that is, the correlation between features is reduced, and the data mean and standard deviation are normalized so that the mean value of each dimensional feature is 0 and the standard deviation is 1. In the actual construction process, we generally place the BN layer between the activation function and the convolution operation, so the forward-conducting convolution calculation equation (4) is transformed as follows:

(5) $$\begin{array}{c} x_{j^{\prime }}^{l}=f\left(\mathrm{BN}\left(\sum_{j\in M^{l}}x_{j}^{l-1}*f_{jj^{\prime }}^{l}\right)\right). \end{array}$$

The pooling layer is to downsample the feature map of the previous convolutional layer to obtain a smaller-dimensional output feature map that corresponds to the input feature map one to one.

(6) $$\begin{array}{c} x_{j^{\prime }}^{l}=f\left(\beta_{j^{\prime }}^{l}\mathrm{down}\left(x_{j^{\prime }}^{l-1}\right)\right), \end{array}$$

where down(·) is the downsampling function and *β* is the downsampling coefficient. Similar to the convolutional layer, on the pooling layer we also normalize the feature map by introducing a BN layer, and its position is generally placed between the activation function and the pooling operation so that the forward-conducting pooling calculation equation (6) is transformed into

(7) $$\begin{array}{c} x_{j^{\prime }}^{l}=f\left(\mathrm{BN}\left(\beta_{j^{\prime }}^{l}\mathrm{down}\left(x_{j^{\prime }}^{l-1}\right)\right)\right). \end{array}$$

The DCN model is trained adopting a backpropagation layer-by-layer training mechanism, and the parameters to be trained are convolutional kernel ***f***. Let ${\hat{y}}_{n}^{\left(i\right)}$ denote the *m*th dimension of the label corresponding to the *i*th sample. *y*_*m*_^(*i*)^ denotes the *m*-dimension of the output corresponding to the *i*th sample. The squared error cost function is

(8) $$\begin{array}{c} J\left(f\right)=\frac{1}{2}\sum_{i=1}^{N}\overset{M}{\underset{m=1}{\sum }}{\left({\hat{y}}_{m}^{\left(i\right)}-y_{m}^{\left(i\right)}\right)}^{2}, \end{array}$$

where *M* denotes the total number of categories. The update formula of the convolution kernel using small batches of stochastic gradient descent is as follows:

(9) $$\begin{array}{c} f_{jj^{\prime }}^{l}\left(t\right)=f_{jj^{\prime }}^{l}\left(t-1\right)-\frac{1}{N}\eta \sum_{i=1}^{N}\frac{\partial J}{\partial f_{jj^{\prime }}^{l}\left(t-1\right)}, \end{array}$$

where *t* denotes the current moment and *η* is the learning rate. It is well known that in the process of training DCN with MB-SGD method, when the gradient keeping direction changes, the error surface has different curvature along different directions, which is easy to cause the points on the surface to oscillate from one side to the other with the continuous descent of gradient so that the gradient cannot converge to the minimum value [30]. Therefore, we consider retaining both the gradient vector information at the last time in the MB-SGD method and the second derivative information of the error function obtained when the network parameters are updated at the last time. This second derivative information estimates not only the gradient of the surface of the cost function at a point (first-order information), but also the curvature of the surface (second-order information). Once the curvature is calculated, the approximate location of the minimum value of the cost function can be estimated. The update formula of the convolution kernel after obtaining the second derivative information is

(10) $$\begin{array}{c} \Delta f_{jj^{\prime }}^{l}\left(t-1\right)=\frac{\nabla f_{jj^{\prime }}^{l}\left(t-1\right)}{\nabla f_{jj^{\prime }}^{l}\left(t-2\right)-\nabla f_{jj^{\prime }}^{l}\left(t-1\right)}\Delta f_{jj^{\prime }}^{l}\left(t-2\right), \end{array}$$

where ∇*f*_*jj* ′_^*l*^(*t* − 1) is the gradient function at moment *t* − 1. From the QuickProp theory proposed by Fahlman [31], it is known that if the step size in the convolutional kernel update formula grows too fast, it tends to cause the convergence process to diverge. Therefore, a momentum factor *µ* is introduced to overcome the aforementioned drawback. Equation (11) is equivalent to equation (12) when the conditions of equation (11) are established.

(11) $$\begin{array}{c} \Delta f_{jj^{\prime }}^{l}\left(t-1\right)>\mu \Delta f_{jj^{\prime }}^{l}\left(t-2\right), \end{array}$$

(12) $$\begin{array}{c} \Delta f_{jj}^{l}\left(t-1\right)=\mu \Delta f_{jj^{\prime }}^{l}\left(t-2\right). \end{array}$$

Based on the above analysis, equation (9) is transformed to

(13) $$\begin{array}{c} f_{jj^{\prime }}^{l}\left(t\right)=f_{jj^{\prime }}^{l}\left(t-1\right)-\frac{1}{N}\eta \sum_{i=1}^{N}\mu \frac{\partial J}{\partial f_{jj^{\prime }}^{l}\left(t-2\right)}. \end{array}$$

The article "Classification of Benign and Malignant Lung Nodules Based on Deep Convolutional Network Feature Extraction" was published in 2021. Journal: J Healthc Eng.

## 3. Results and Discussion

### 3.1. Implementation Details

In this section, the deep network used in the experiments consists of three blocks, each with the same number of layers, including a convolutional layer, a multilayer perceptron layer, and a pooling layer. After the original data is input to the first block, a convolution operation with a step size of 1 and a convolution kernel size of 5 × 5 is performed on the input image to extract features. Then, two perceptron layers with a step size of 1 and a convolution kernel size of 1 × 1 are used to interact and integrate feature information. Finally, a pooling layer with a size of 2 × 2 and a step size of 2 is used to downsample. The first pooling layer uses a maxpool and the rest uses an averagepool. At the end of the last block, a softmax-loss classifier is attached after the averagepool is executed. The feature mapping dimensions in the three blocks are 28 × 28, 12 × 12, and 4 × 4, respectively. The exact network configuration we use on the dataset is shown in Table 1.

### 3.2. Training Setup

We use a MATLAB-based deep learning framework (MatConvNet) for the construction of the proposed deep network model on a workstation with a Win10 system, i9 processor, and 64G RAM. We choose stratified 10-fold cross-validation as a rigorous validation model [20]. All data is randomly divided into 10 subsets. Nine of these subsets were used for training and one for testing, which was repeated ten times. In the training stage, we used the MB-SGD method to optimize the model. We initialize the parameters according to our experience. The initial learning rate is set 0.1, and the minibatch size is 50. We adopt the weight initialization strategy described in [32] with a weight decay of 0.0001. Our experiments had carried out a total of 120 epochs.

### 3.3. Validation of Hyperparameter

In this paper, we need to modify the proposed network parameters repeatedly by using the method of MB-SGD and finally make the result of the loss function reach the minimum value. For the MB-SGD method with a momentum coefficient, the value of the momentum coefficient *μ* directly affects the location of the minimum cost function, which in turn affects the classification accuracy of the lung nodule images. For this reason, it is necessary to discuss the value of *μ*. According to the description in the training setup, ten experiments with 10 different values of *μ* were conducted to select the best value. We change the value of *μ* from 0 to 1 at intervals of 0.1.  Table 2 shows the impact of different *μ* values on model classification performance. It can be seen that the classification error rate of lung nodule images gradually decreased as the value of *μ* increases. When *μ* is 0.9, the model can obtain the lowest classification error rate.

### 3.4. Empirical Study

#### 3.4.1. Classification of Benign and Malignant Lung Nodules under Different Sample Configuration Schemes

In this section, we conduct a series of experiments to find the most suitable sample configuration scheme. According to the data distribution method in the training set, a subset (75 samples) is randomly selected as the testing set. To verify the impact of the training set size on the generalization abilities of the model, we gradually increase the size of the training samples. As can be seen from the result in Figure 3, changing the size of the training samples has an impact on the classification performance of the network. As the number of training samples increases, network classification accuracy tends to increase. When the training samples are 500 or 550, our network model achieves the best classification performance. After that, the network classification performance shows a decreasing trend. This problem may be limited by the size of the number of cases in the dataset and the disappearance of a gradient.

The article "Classification of Benign and Malignant Lung Nodules Based on Deep Convolutional Network Feature Extraction" was published in 2021. Journal: J Healthc Eng.

#### 3.4.2. Optimizer Selection

Gradient descent algorithm is the most commonly used optimization method in machine learning, and current networks are trained using different gradient descent algorithms for network training. Therefore, a good optimizer design in practical applications is of great importance to avoid the gradient dispersion of the deep network. In this section, to test the speed and stability of the proposed MB-SGD method with momentum coefficients during the training process, we plot the RL curves and analyze the effectiveness of the proposed algorithm by comparing it with the traditional MB-SGD method. The mean square error RL curve is a smoothing sequence with minimum mean square error, and its shape shows that with the increase of the number of iterations, the CNN model training process predicts the error. On the other hand, it also represents the speed and stability of the network convergence. In this experiment, the minibatch size is 50 and the training samples are 500. After training the sample data once, the weights are iteratively updated 10 times, and after performing 120 epochs of training, the weights are iteratively updated 1200 times. The experimental results are shown in Figure 4. It can be seen that the two learning algorithms have similar minimum mean square error values in the initial phase of training. With the increase of the number of iterations, the RL curves of both algorithms show a gradual decrease, which indicates that the training network is stable and reliable. It is worth noting that the RL curve of MB-SGD shows a smooth trend from the 200th iteration to the 700th iteration. In addition, the MB-SGD with a momentum coefficient has smaller minimum mean square error values than the MB-SGD. This indicates that MB-SGD with a momentum coefficient has faster and more stable convergence during network training.

#### 3.4.3. Deep Network Architecture Comparison

One of the most important advantages of deep learning is the ability to automatically learn relevant features from the original image. To further evaluate the effectiveness of the proposed method, classical deep learning models such as CNN, DBN, and SAE were used to extract lung nodule features and perform classification experiments under the same dataset segmentation.  Table 3 gives a comparison of the classification results under different deep learning models. It can be seen that our proposed DCN model obtains superior classification performance compared to other deep learning classical models. In addition, in the classic deep learning model, the classification performance of CNN is better than that of DBN and SAE.  Figure 5 shows the visualization of the lung nodule features extracted by the three deep learning classical models. The results show that the feature visualization results extracted by CNN are more abstract. Meanwhile, combined with the experimental results in Table 3, it can be seen that CNN has obvious advantages in image feature extraction.

The article "Classification of Benign and Malignant Lung Nodules Based on Deep Convolutional Network Feature Extraction" was published in 2021. Journal: J Healthc Eng.

#### 3.4.4. Results' Analysis

To highlight the performance of our proposed method, we compared our results with those of the literature designed for lung nodule classification. As shown in Table 4, all methods used the LIDC database for experiments. In this study, because these nodules lack the results of histopathology, and the small size of lung nodules, it is unrealistic to classify lung nodules by processing the whole image. Therefore, all methods extract the lung nodule area based on the nodule center coordinates marked by the doctor in the XML file, and process the data according to the proposed method. Finally, according to the proposed model, different numbers and types of lung nodule samples were obtained. It can be seen from Table 4, compared with 2D-CNN [4, 33–35], 3D-CNN [20, 21, 36] achieves better classification performance while using fewer lung nodule samples. This is mainly because 3D-CNN can extract spatial information from lung nodules more effectively. The results show that our proposed method outperforms the other existing works, and it also proves the effectiveness of the proposed DCN with MB-SGD for the classification of lung nodules. Moreover, compared with a single CNN classification model, a model that combines different classifiers and features fusion has better classification performance. In addition, this study has also demonstrated the importance of the process that we must choose to improve the performance of the model.

## 4. Conclusions

As one of the most popular research directions in the field of machine learning, deep learning can learn advanced features of data and has more powerful nonlinear representation capabilities. In this study, we propose a novel DCN learning method for the benign and malignant classification of lung nodules. The main advantages are as follows: (1) perform ZCA whitening processing on the extracted lung nodule images, which can effectively eliminate redundant information between pixels; (2) combine the multilayer perceptron layer with CNN to construct a DCN model capable of learning strongly robust features, thus improving the feature representation power of the network to a greater extent; (3) the MB-SGD method with a momentum coefficient is used to train the deep network, which effectively avoids the local optimum and gradient dispersion phenomena. The experimental results on the LIDC dataset show that the proposed DCN learning method has high classification accuracy for benign and malignant classification of lung nodules.

The article "Classification of Benign and Malignant Lung Nodules Based on Deep Convolutional Network Feature Extraction" was published in 2021. Journal: J Healthc Eng.

## Figures and Tables

**Figure 1:** Schematic diagram of the benign and malignant lung nodules' classification system based on DCN feature extraction.

**Figure 2:** The processed part of the sample images of lung nodules.

**Figure 3:** Classification accuracy under different sample configuration schemes.

**Figure 4:** The convergence process of the DCN structure in the process of training. (a) MB-SGD. (b) MB-SGD with momentum coefficient.

**Figure 5:** Visual display of classical deep learning model feature extraction. (a) CNN. (b) DBN. (c) SAE.

**Table 1:** Network parameter configuration.

Layers	Input			Kernel number	Kernel size	Stride	Pad	Output		
	W	H	D					W	H	D
Input								28	28	1
conv1	28	28	1	6	5	1	0	24	24	6
cccp1	24	24	6	6	1	1	0	24	24	6
cccp2	24	24	6	6	1	1	0	24	24	6
maxpool1	24	24	6		2	2	0	12	12	6
conv2	12	12	6	12	5	1	0	8	8	12
cccp3	8	8	12	12	1	1	0	8	8	12
cccp4	8	8	12	12	1	1	0	8	8	12
avgpool2	8	8	12		2	2	0	4	4	12
conv3	4	4	24	24	4	1	0	1	1	24
cccp5	1	1	24	24	1	1	0	1	1	24
cccp6	1	1	24	2	1	1	0	1	1	2
Avgpool3	1	1	2		2	2	0	1	1	2
Softmax-loss	1	1	2					1	1	2

**Table 2:** The impact of different *μ* values on model classification performance.

	*μ* = 0.1	*μ* = 0.2	*μ* = 0.3	*μ* = 0.4	*μ* = 0.5
Error (%)	11.5	11.0	10.9	9.6	9.1
	*μ* = 0.6	*μ* = 0.7	*μ* = 0.8	*μ* = 0.9	*μ* = 1
Error (%)	9.0	8.4	8.0	7.5	11.4

**Table 3:** Comparison of classification results of different DL architectures.

Method	Error (%)
DCN	4.0
CNN	19.15
DBN	20.58
SAE	21.43

**Table 4:** Comparison of the results of different methods.

Method	Number of nodules	Error (%)
Multiscale CNN [33]	865	15.9
AlexNet + cascaded classifier [34]	1990	15.3
VGG16 + SVM [35]	1945	12.2
B-CNN-FT [4]	3186	8.8
3D-CNN + QIF [36]	664	6.8
3D-CNN + multiscale + multi [20]	962	6.08
3D-Inception-ResNet + hand-crafted features [21]	1036	5.02
DCN + MB-SGD	750	4.0

## Data Availability

The data used to support the findings of this study are available from the first author upon request.
